The article "Computed Tomography Image under Convolutional Neural Network Deep Learning Algorithm in Pulmonary Nodule Detection and Lung Function Examination" was published in 2021. Journal: J Healthc Eng.

# Computed Tomography Image under Convolutional Neural Network Deep Learning Algorithm in Pulmonary Nodule Detection and Lung Function Examination

**DOI:** 10.1155/2021/3417285

**Published:** 2021-10-22

**Authors:** Chan Zhang, Jing Li, Jian Huang, Shangjie Wu

**Affiliations:** ^1^Department of Respiratory Medicine, Xiangya Second Hospital of Central South University, Changsha 410006, Hunan, China; ^2^Department of Imaging, Changsha Fourth Hospital (Changsha Hospital Affiliated to Hunan Normal University), Changsha 410006, Hunan, China

## Abstract

The objective of this study was to perform segmentation and extraction of CT images of pulmonary nodules based on convolutional neural networks (CNNs). The Mask-RCNN algorithm model is a typical end-to-end image segmentation model, which uses the R-FCN structure for nodule detection. The effect of applying the two algorithm models to the computed tomography (CT) diagnosis of pulmonary nodules was analyzed, and different indexes of pulmonary nodule CT images in lung function examination after algorithm optimization were compared. A total of 56 patients diagnosed with pulmonary nodules by surgery or puncture were taken as the research objects. Based on the Mask-RCNN algorithm, a model for CT image segmentation processing of pulmonary nodules was proposed. Subsequently, the 3D Faster-RCNN model was used to label the nodules in the pulmonary nodules. The experimental results showed that the trained Mask-RCNN algorithm model can effectively complete the segmentation task of lung CT images, but there was a little jitter at the boundary. The speed of R-FCN algorithm for nodular detection was 0.172 seconds/picture, and the accuracy was 88.9%. CT scans were performed on the 56 patients based on a deep learning algorithm. The results showed that 30 cases of malignant pulmonary nodules were confirmed, and the diagnostic accuracy was 93.75%. There were 22 benign lesions, the diagnostic accuracy was 91.67%, and the overall diagnostic accuracy was 92.85%. This study effectively improved the diagnostic efficiency of CT images of pulmonary nodules, and the accuracy of CT images in the diagnosis of pulmonary nodules was analyzed and evaluated. It provided theoretical support for the follow-up diagnosis of pulmonary nodules and the treatment of lung cancer. It also significantly improved the diagnostic effect and detection efficiency of pulmonary nodules.

## 1. Introduction

Pulmonary nodules are considered to be a multi-system and multi-organ granulomatous disease with unknown etiology at present, which often occurs in the lungs, bilateral hilar lymph nodes, eyes, skin, and other organs, and the incidence in the chest is as high as 80%–90% [1]. At present, there have been many studies on the pathogenic causes of pulmonary nodules, including observation and study on bacteria, viruses, mycoplasma, fungi, and other infectious factors, but the exact pathogenic causes have not been obtained. According to relevant studies, most people currently believe that the important pathogenesis of pulmonary sarcoidosis is the disorder of cellular immune function and humoral immune function, which is the result of the interaction between cellular immunity and humoral function of the body caused by unknown antigens [2, 3]. In recent years, with the development of society and changes of environment, the incidence of various lung diseases in China has been on the rise, among which lung cancer has become the cancer with the highest incidence in China. According to relevant data [4], in 2015 alone, the number of deaths due to lung cancer in China reached more than 700,000. Lung cancer was the leading cause of cancer deaths in 2018, accounting for 20 percent of all cancer deaths. By the end of 2017, the number of lung cancer patients and deaths in China had reached 800,000 and 700,000. The incidence of lung cancer is increasing at an annual rate of 27%, based on which the mortality rate of lung cancer patients in China will increase to 40% in the next 20 years [5].

The article "Computed Tomography Image under Convolutional Neural Network Deep Learning Algorithm in Pulmonary Nodule Detection and Lung Function Examination" was published in 2021. Journal: J Healthc Eng.

The manifestations of early lung cancer are mainly pulmonary nodules, and there are generally no other specific symptoms in clinical practice. Lung cancer usually goes undetected by patients until they have obvious symptoms. Such symptoms include fever caused by repeated infection, inflammation of the lungs, chest tightness and shortness of breath, persistent coughing and hemoptysis, and excessive fatigue. At that time, lung cancer has generally entered the middle and late stages, and the best treatment period has been missed. At this time, the optimal treatment period has been missed, so the early diagnosis of lung cancer is extremely important. One of the key factors determining the survival rate of patients with lung cancer is the early accurate diagnosis of pulmonary nodules [6, 7]. If early pulmonary nodules are diagnosed and treated in advance and its early symptoms and related indicators are studied, it can effectively improve the early diagnosis rate and survival rate of lung cancer patients.

Currently, the main detection methods for lung cancer include computed tomography (CT) [1, 8]. CT is based on X-ray technology. The X-ray is sent out by the scanner in a fan-shaped wire bundle of a certain thickness to illuminate the patient at different angles. Then, the collected data are converted into current intensity signals in and out of the computer through the scanner and finally converted into three-dimensional images through the algorithm. CT detection is very important in the examination of lung function, but the analysis and diagnosis of lung CT images are often affected by doctors' experience and other subjective reasons. The diagnosis of the same CT image varies greatly among doctors of different skills, and a large number of CT images also produce excessive burden on radiologists. Therefore, algorithm-assisted processing of CT images based on convolutional neural network (CNN) is extremely important. Generally, there are two important methods for the algorithm-assisted CT diagnosis of pulmonary nodules [9, 10]. The first is the segmentation of lung CT images. To ensure that doctors can observe the nodules in the three-dimensional images carefully, the lung parenchyma needs to be segmented to remove the irrelevant data in the CT images. The second is adopting the algorithm to automate the detection of pulmonary nodules in CT images, which can not only effectively improve the diagnostic efficiency of radiologists but also improve the poor diagnostic effect caused by subjective differences.

The article "Computed Tomography Image under Convolutional Neural Network Deep Learning Algorithm in Pulmonary Nodule Detection and Lung Function Examination" was published in 2021. Journal: J Healthc Eng.

Therefore, a model for CT image analysis of pulmonary nodules was proposed based on CNN deep learning technology, and then a comparison of different indexes of lung function examination of pulmonary nodules CT images was conducted after the optimization of the algorithm. The results of this study were intended to provide reference for the improvement of clinical diagnosis and treatment of patients with pulmonary nodules.

## 2. Methods

### 2.1. Research Objects

Fifty-six patients with pulmonary nodules confirmed by surgery or puncture in the hospital from May 2018 to May 2020 were selected as the research subjects. All patients received CT and MRI examination at admission and had complete clinical diagnosis records and imaging data. Among the 56 patients, 34 were males and 22 were females. Patients ranged in age from 30 to 77 years, with a mean age of (56.8 ± 4.7) years. The diameter of nodules in all patients ranged from 1.1 cm to 2.8 cm, with an average diameter of (2.0 ± 0.4) cm. There were 28 cases of right pulmonary nodules and 27 cases of left pulmonary nodules. All patients had signed informed consent, and this study had been approved by the Ethics Committee of the hospital.

Inclusion criteria were as follows: (i) those who met the diagnostic criteria of pulmonary nodules; (ii) patients who did not receive any radiotherapy, chemotherapy, or other treatment before treatment; (iii) patients who had no other serious heart, liver, kidney, and brain diseases or malignant tumors; (iv) patients who agreed and accepted the research; and (v) patients who were not allergic to contrast agents.

The article "Computed Tomography Image under Convolutional Neural Network Deep Learning Algorithm in Pulmonary Nodule Detection and Lung Function Examination" was published in 2021. Journal: J Healthc Eng.

Exclusion criteria were as follows: (i) patients with imperfect imaging data; (ii) patients who were unable to cooperate with the completion of imaging examination; (iii) patients who were allergic to contrast agents; and (iv) patients with other serious heart, liver, kidney, and brain diseases or malignant tumors.

### 2.2. CT Examination

Whole-body low-dose CT was performed using a Siemens Somatom Emotion 16-slice spiral CT scanner. Patients were trained to hold their breath before the scan, and the whole lung scan was performed. Voltage and current were set as 120 kV and 100 mAs, respectively. The layer thickness was 8.0 mm, layer spacing was 1 mm, reconstruction interval was 8.0 mm, pitch was 0.811, and collimation was 16 × 0.75. For a CT scan, the patient was supine with arms crossed and placed in the lower abdomen. During scanning, the maximum layer of pulmonary nodules was selected for dynamic enhanced scanning. After the scanning range was reduced, the nonionic contrast agent ioversol (320 mgl/mL) was injected through cubital vein with high pressure, the dose was 90 mL, and the rate was 4.0 mL/s.

### 2.3. CT Image Segmentation Based on Mask-RCNN Algorithm Model

The Mask-RCNN algorithm model is a type of algorithm that combines detection and classification based on the Faster-RCNN algorithm. It is a convolutional neural network model that combines object detection and image segmentation [11]. Under the interaction of the target detection algorithm and the segmentation algorithm, the pixel-level segmentation effect is achieved, and the segmentation of the CT image is completed efficiently and quickly. Unlike the Faster-RCNN algorithm, the Mask-RCNN algorithm replaces the ROI pooling layer in the original algorithm with a better ROI alignment layer, which effectively improves the accuracy of the image segmentation boundary [12]. Based on the new network model, a fully convolutional network is used for image segmentation. The structure diagram is shown in Figure 1.

The change of the ROI alignment layer is the most important update implemented on the Mask-RCNN algorithm repooling layer, which realizes the mutual correspondence between output pixels and input pixels and effectively retains the spatial data contained in the image. The target pixel position in the original CT image in the image processing process is calculated by the following equations.

(1) $$\begin{array}{c} \text{Src}M=\text{dst }M\left(\frac{\text{src Width}}{\text{dst Width}}\right),\\ \text{Src}N=\text{dst }N\left(\frac{\text{src Height}}{\text{dst Height}}\right), \end{array}$$

where dstM and dstN represent the pixel coordinates in the area suggestion box, srcM and srcN represent the coordinates of the target pixel in the original CT image, srcWidth and srcHeight represent the width and height of the original image, respectively, and dstWidth and dstHeight are the width and height of the regional suggestion box, respectively. The following equation is used to calculate the pixel value of the sampling point of each unit through the bilinear interpolation method, and then the maximum pooling operation is implemented.

(2) $$\begin{array}{c} t\left(e+f,g+h\right)=\left(1-f\right)\left(1-h\right)t\left(e,g\right)+\left(1-f\right)ht\left(e,g+1\right)+f\left(1-h\right)+\left(e+1,g\right)+fht\left(e+1,g+1\right). \end{array}$$

In the equation, there are four coordinate points to interpolate the *M* and *N* directions.

The article "Computed Tomography Image under Convolutional Neural Network Deep Learning Algorithm in Pulmonary Nodule Detection and Lung Function Examination" was published in 2021. Journal: J Healthc Eng.

The loss function is used to train the model, which includes the bounding box regression loss and the target classification loss. The overall loss function expression equation is as follows.

(3) $$\begin{array}{c} k=k_{clS}+k_{\text{box}}+k_{\text{mask}}, \end{array}$$

where *k*_mask_ refers to the average binary cross-entropy loss, and its expression is as follows.

(4) $$\begin{array}{c} \text{Crossentropy}\left(t,0\right)=-\left(t,\;\log\left(v\right)+\left(1-t\right)\log\left(1-v\right)\right), \end{array}$$

where *t* represents the target and *v* represents the output of the network model. The processing of the loss function generates labels of different category attributes for objects of different categories so that the interaction between the same categories will not occur.

### 2.4. Pulmonary Nodule Detection Algorithm Based on R-FCN

The CT image of the lungs segmented by the Mask-RCNN algorithm was used as the input of CNN for feature extraction. Subsequently, the fully convolutional network R-FCN was used as the detection algorithm model for pulmonary nodules, which is an end-to-end network model [13]. Similar to Faster-RCNN, R-FCN also performs network extraction of ROI, but Faster-RCNN loses certain characteristics after the extraction process. To retain some of the missing features, Faster-RCNN uses a deeper network model, but it undoubtedly sacrifices the training and testing efficiency of the model. The R-FCN used encodes location information by creating a location-sensitive feature map to retain the relevant features of the data, and there is no convolutional layer behind the pooling layer. The model's structure and location-sensitive features are shown in Figures 2 and 3.

For the grid of the *m*th row and *n*th column of the target object *F*, the expression of the position-sensitive pooling layer is as follows.

(5) $$\begin{array}{c} r_{F}\left(m,n\;|\;\theta \right)=\sum_{\left(x,y\right)\varepsilon \text{bin}\left(m,n\right)}\frac{z_{m,n,F}\left(x+x_{0},y+{y_{0}\;|\;}_{\theta }\right)}{n}, \end{array}$$

where *r*_*F*_(*m*, *n*) represents the average score of the (*m*, *n*)th network in the *F* target after passing through the pooling layer, *z*_*m*,*n*,*F*_ is an output of the sensitive feature map at the *k*^2^(*F*+1)th position, (*x*_0_, *y*_0_) represents the coordinates of the ROI, *n* means the number of all pixels in the model, and *θ* represents the parameters in the network; the score expression of the target *F* object is as follows.

(6) $$\begin{array}{c} r_{F}\left(\theta \right)=\sum_{m,n}r_{F}\left(m,n\;|\;\theta \right). \end{array}$$

Then, the loss function of each target object consisting of cross-entropy loss and boundary regression loss is calculated.

(7) $$\begin{array}{c} k\left(r,v_{x,y,w,h}\right)=K_{c_{l}s}\left(r_{c^{*}}\right)+\phi \left[c^{*}>0\right]k_{\text{reg}}\left(v,v^{*}\right), \end{array}$$

where *c*^∗^ represents the true calibration value of ROI, *K*_*c*_*l*_*s*_(*r*_*c*^*∗*^_) represents the cross-entropy loss function, *k*_reg_(*v*, *v*^*∗*^) represents the boundary loss function, and *v*^*∗*^ represents the real border of the ROI.

The article "Computed Tomography Image under Convolutional Neural Network Deep Learning Algorithm in Pulmonary Nodule Detection and Lung Function Examination" was published in 2021. Journal: J Healthc Eng.

### 2.5. Statistical Mathematical Processing

SPSS 19.0 was used for statistical analysis. The measurement data conforming to normal distribution were expressed as mean ± standard deviation, and the difference between groups was analyzed by independent sample *t*-test. The measurement data that did not conform to normal distribution were represented by median value and quad position, and the comparison between groups was analyzed by nonparametric rank sum test. *N* (%) was used to represent the count data, and chi-square test was used to analyze the difference between groups. The *p* value was calculated according to the variance value, and *p* < 0.05 was considered statistically significant.

## 3. Results

### 3.1. Image Segmentation Results Based on Mask-RCNN Algorithm Model

The deep learning framework for algorithm models was TensorFlow. This learning framework has a high degree of flexibility and strong portability, which supports multi-language and automatic differentiation. Regarding the training of the algorithm model, the CT image data used in this study were all the medical image data of the observation objects selected.

The training of the Mask-RCNN algorithm model used a stochastic gradient descent training network (SGD), the number of iterations (epoch) was 500, the momentum was 0.8, the learning rate was 0.0001, the batch size was 4, and the weight attenuation was 0.0001. After 400 iterations of the network model, the loss started to converge. Therefore, it was decided to use the training model after 450 iterations to segment the lung CT image. The comparison chart of the effect before and after segmentation is shown in Figure 4.

The article "Computed Tomography Image under Convolutional Neural Network Deep Learning Algorithm in Pulmonary Nodule Detection and Lung Function Examination" was published in 2021. Journal: J Healthc Eng.

From the before and after comparison of the segmentation effect of the Mask-RCNN algorithm model on the lung CT image, the trained Mask-RCNN algorithm model can effectively complete the segmentation task of the lung CT image, but there was a slight jitter at the boundary. Therefore, the Mask-RCNN algorithm model cannot fully learn the boundary features of the image, but the segmentation of the lung parenchyma fully met the requirements.

### 3.2. Comparison of Results of Pulmonary Nodule Detection Algorithms Based on R-FCN

The CT image data used in this section were all the medical image data of the observed objects selected in this study. Each lung CT image contained pulmonary nodules with a diameter range of approximately 1.1 cm–2.8 cm, with an average diameter of (2.0 ± 0.4) cm. The position and shape of nodules in all CT images were not fixed. Randomly assigned according to a 2 : 1 ratio, the datasets were divided into training set and verification set. Nodules on all CT images contained both benign and malignant lesions. Malignant lesions were characterized by irregular and burr-like edges and exponential growth rate. Benign lesions were characterized by nodules with relatively smooth edges and slow growth.

The training of the R-FCN algorithm model used a stochastic gradient descent training network (SGD), the number of iterations (epoch) was 500, the momentum was 0.8, the learning rate was 0.0001, the batch size was 4, and the weight decay was 0.0001. According to the experimental results, the speed of R-FCN algorithm for nodule detection was 0.172 seconds/frame, and the accuracy was 88.9%. The results before and after the test are shown in Figure 5.

### 3.3. CT Image Performance of Different Pulmonary Nodules Based on Deep Learning

Fifty-six patients who were diagnosed with pulmonary nodules by surgery or puncture in the hospital in a certain area were the research objects. Among 56 cases of pulmonary nodules diagnosed after surgery or pathological examination, 32 cases were malignant lesions and 24 cases were benign lesions. CT scans based on deep learning algorithms were performed on these 56 patients, 30 cases of malignant lesions of pulmonary nodules were confirmed, and the diagnosis accuracy was 93.75%. There were 22 cases of benign lesions, the diagnostic accuracy was 91.67%, and the overall diagnostic accuracy was 92.85%. At the same time, MRI scan diagnosis was performed, 27 cases of malignant lesions were detected, and the diagnosis accuracy was 84.38%. 16 cases of benign lesions were detected, the diagnostic accuracy was 66.66%, and the overall diagnostic accuracy was 76.78%. In Figure 6, the accuracy of CT scan based on deep learning for the diagnosis of pulmonary nodules was higher than that of MRI.

The article "Computed Tomography Image under Convolutional Neural Network Deep Learning Algorithm in Pulmonary Nodule Detection and Lung Function Examination" was published in 2021. Journal: J Healthc Eng.

The CT scan parameters of different pulmonary nodules were recorded. The peak enhancement (PH) and the ratio of aortic enhancement (SPH/PPH) of malignant nodules and inflammatory nodules were higher than those of benign nodules. The detailed values are shown in Figures 7–8.

## 4. Discussion

The incidence of lung diseases has been increasing year by year, and lung cancer has become the number one enemy affecting the health of Chinese people in recent years. As an important feature of early lung cancer, pulmonary nodules are of great significance for the medical diagnosis and observation analysis of lung cancer. Rapid and effective diagnosis of pulmonary nodules can effectively improve the survival rate of patients with pulmonary diseases.

In the current clinical diagnosis of pulmonary nodules, it is generally believed that benign pulmonary nodules mainly occur in the posterior part of the upper lobe and the dorsal part of the lower lobe of the lung [14–16]. Most of the inflammatory nodules were found in the dorsal and inferior lobes of the lungs. The common sites of malignant nodules are mainly the upper lobe, lingual lobe, and middle lobe of the lung. The morphology of pulmonary nodules is classified into lobular, quasi-circular, and irregular shapes. The quasi-round shape is mainly manifested by the accumulation of nodular masses, usually with expansible growth, and malignant and benign can occur. The irregularity is usually seen in inflammatory nodules. The lobulated nodules are characterized by oval or round mass with uneven surface. According to relevant data, lobulated nodules are present in more than 70% of lung cancer patients [17]. Malicious nodules often have lobulated contours or irregular nodular edges. Almost 90% of lobulated nodules are malignant lesions. Malignant nodules also have features other than lobulated nodules, such as burr-like features, pleural depression, and obvious fibrous tissue proliferation in and around the nodules.

At the present stage of clinical treatment, fiberoptic bronchoscopy, CT, MRI, and needle biopsy are all conventional methods for the diagnosis of pulmonary nodules. However, due to the low sensitivity and limited value of chest radiograph, fiberoptic bronchoscopy has been gradually phased out in the diagnosis of early lung cancer [18]. In addition, puncture biopsy is an invasive operation for tumor detection, which will cause certain physical and mental damage to patients and has poor tolerance. The spatial resolution of MRI imaging examination is low [19], and the morphological characteristics of small and medium-sized pulmonary nodules are not obvious. Moreover, the price is relatively high. CT is currently a research hotspot in the examination of pulmonary nodules, with its remarkable advantages of fast and efficient scanning, small noninvasive radiation, and high tissue resolution. It can not only provide the morphological information of pulmonary nodules but also have a good display rate of the subtle signs of pulmonary nodules.

The article "Computed Tomography Image under Convolutional Neural Network Deep Learning Algorithm in Pulmonary Nodule Detection and Lung Function Examination" was published in 2021. Journal: J Healthc Eng.

At present, CT images have become one of the procedures of routine clinical examination, and the number of CT images has increased greatly in recent years, which has certain requirements on the diagnostic accuracy and efficiency of radiologists. Therefore, it is of great significance to help radiologists effectively improve the diagnostic efficiency. Nowadays, CT scanning equipment has high spatial resolution [20, 21]. With the gradual development of computer and artificial intelligence algorithms, the automation engineering in the field of medical imaging has become increasingly important. Deep learning algorithms have been widely used in image processing, such as image segmentation, target selection, and image enhancement [22, 23]. In today's environment of significantly enhanced server computing capacity, richer datasets, and perfect network training technology, many algorithm models have been proposed. The recognition ability and precision of medical images are also gradually improving. When applied to the processing of medical images, it can completely replace doctors' preliminary subjective diagnosis of diseases in some cases.

## 5. Conclusion

This study aimed to use deep learning technology to segment and extract the CT images of pulmonary nodules, so as to further improve the clinical diagnosis effect of pulmonary nodules. The results showed that the speed of R-FCN algorithm for nodule detection was 0.172 seconds/piece, and the accuracy was 88.9%. By comparing the CT image effects after segmentation detection, the diagnostic accuracy of CT scan based on deep learning for pulmonary nodules was 91.67%, and the overall diagnostic accuracy was 92.85%. CT scan parameters of pulmonary nodules with different properties were recorded. The enhancement peak value (PH) and aortic enhancement value ratio (SPH/PPH) of malignant and inflammatory nodules were higher than those of benign nodules, and the data showed good consistency with the results of surgical examination. Moreover, the data showed a good agreement with the results of surgical examination. These results indicated that CT images based on deep learning were efficient and accurate in the diagnosis of pulmonary nodules. However, the research content of this work still has some limitations. Only a single imaging diagnosis method was studied, and the sample size was not large enough. At present, only automatic detection and labeling of pulmonary nodules can be achieved, but the nature of nodules cannot be distinguished, and artificial diagnosis is still needed. Therefore, it is necessary to increase the number of samples and further explore the deep learning algorithm in the future. In conclusion, this study can effectively improve the diagnostic efficiency of CT images for pulmonary nodules, and analyze and evaluate the accuracy of CT images for pulmonary nodules. In addition, it provides theoretical support for the follow-up diagnosis of pulmonary nodules and the treatment of lung cancer and also significantly improves the diagnostic effect and detection efficiency of pulmonary nodules.

The article "Computed Tomography Image under Convolutional Neural Network Deep Learning Algorithm in Pulmonary Nodule Detection and Lung Function Examination" was published in 2021. Journal: J Healthc Eng.

## Figures and Tables

**Figure 1:** Schematic diagram of Mask-RCNN algorithm segmentation.

**Figure 2:** Schematic diagram of R-FCN model structure.

**Figure 3:** Location-sensitive feature map of R-FCN.

**Figure 4:** Comparison of the segmentation effect of Mask-RCNN algorithm on lung CT images (the box represents the automatic selection and labeling of lung parenchyma by Mask-RCNN algorithm, and the dotted line represents the further automatic segmentation of lung parenchyma).

**Figure 5:** Comparison of the detection effect of R-FCN algorithm on CT images of pulmonary nodules (the box represents the automatic segmentation labeling of pulmonary nodules by R-FCN algorithm).

**Figure 6:** Comparison of the diagnostic accuracy of CT and MRI on CT images of pulmonary nodules.

**Figure 7:** Enhanced peak CT scan parameters of different types of pulmonary nodules.

**Figure 8:** CT scan parameters of the ratio of aortic enhancement value of different pulmonary nodules.

## Data Availability

The data used to support the findings of this study are available from the corresponding author upon request.
